# A Study of the Brain Network Connectivity in Visual-Word Pairing Associative Learning and Episodic Memory Reactivating Task

**DOI:** 10.1155/2021/5579888

**Published:** 2021-07-08

**Authors:** Mingxin Zhang, Feng Duan, Shan Wang, Kai Zhang, Xuyi Chen, Zhe Sun

**Affiliations:** ^1^College of Artificial Intelligence, Nankai University, No. 38 Tongyan Road, Jinnan District, Tianjin 300350, China; ^2^Department of Surgery, First Teaching Hospital of Tianjin University of Traditional Chinese Medicine, No. 88 Changling Road, Xiqing District, Tianjin 300381, China; ^3^Brain Center, The Hospital of Pingjin, No. 220 Chenglin Road, Hedong District, Tianjin 300162, China; ^4^Computational Engineering Applications Unit, Head Office for Information Systems and Cybersecurity, RIKEN, Wako-Shi, Japan

## Abstract

Episodic memory allows a person to recall and mentally reexperience specific episodes from one's personal past. Studies of episodic memory are of great significance for the diagnosis and the exploration of the mechanism of memory generation. Most of the current studies focus on certain brain regions and pay less attention to the interrelationship between multiple brain regions. To explore the interrelationship in the brain network, we use an open fMRI dataset to construct the brain functional connectivity and effective connectivity network. We establish a binary directed network of the memory when it is reactivated. The binary directed network shows that the occipital lobe and parietal lobe have the most causal connections. The number of edges starting from the superior parietal lobule is the highest, with 49 edges, and 31 of which are connected to the occipital cortex. This means that the interaction between the superior parietal lobule and the occipital lobe plays the most important role in episodic memory, and the superior parietal lobule plays a more causal role in causality. In addition, memory regions such as the precuneus and fusiform also have some edges. The results show that the posterior parietal cortex plays an important role of hub node in the episodic memory network. From the brain network model, more information can be obtained, which is conducive to exploring the brain's changing pattern in the whole memory process.

## 1. Introduction

Episodic memory is the memory for specific events [1]. When two events occur at the same time, the brain will establish a connection between the memories of the two events to form an association. When the memory of one of the events is reactivated, the memory associated with the other event may also be activated again. Studies of generation mechanism of this memory have important practical sense. For example, stimulation over network related to episodic memory can promote the consolidation of memory in older adults [1]. This has a positive effect on the study of phenomena such as memory decline in the elderly [2]. In addition, episodic memory also provides enlightenment for diagnosis and pathology research. The study of the episodic memory phase could help to accurately describe the symptomatic phase of Alzheimer's disease (AD), which could lead to improved treatment regimens [3]. Episodic memory network and hippocampus are also thought to be closely related to Parkinson's disease (PD) [4]. Episodic memory may also aid the diagnosis of other mental disorders such as autism and schizophrenia [5, 6].

Episodic memory is concerned with the storage and retrieval of some events about personal experience, as well as the spatial-temporal relationships between these events [7]. Tulving described it as when recalling an event, people seem to be taken back to the scene of the event, and thus, the cortex involved in the memory retrieval process is reactivated [7]. Current research studies reveal that episodic memory is influenced by interactions between multiple brain regions.

Prefrontal cortex may play an important role on episodic memory. Stimulation to the lateral prefrontal cortex can consolidate episodic memory, while stimulation to the posterior parietal cortex has no obvious effect [8, 9]. There are also some studies working on other memory-related functional networks. A study focus on the connection of the hippocampal-cortical network (HCN) shows a causal relationship in episodic memory retrieval [10]. According to other results of fMRI studies related to memory retrieval, brain regions related to episodic memory are also widely distributed in the temporal, parietal, occipital, frontal, and other regions. Associative stimuli can consolidate the activation intensity of memory. In a learning and test task, a large number of associative stimuli can make the learned word items get stronger activation [11]. Studies have shown that the prefrontal cortex and the medial temporal lobe interaction play an important role in episodic memory. At the same time, the encoding and retrieval of episodic memory is related to the activation of the temporal lobe, prefrontal lobe, and parietal lobe. The upper and dorsal parietal lobes, as well as the anterior prefrontal region, are more active in the retrieval of episodic memory [12]. In addition, some studies have shown that the hippocampus and striatum have strong functional connectivity during associative memory [13]. Also, in addition to some studies focus on the activation of brain regions, there are also studies that attempt to use some machine learning methods to classify fMRI data with different activation patterns [14].

Brain networks related to episodic memory are widely connected, and under different task modes, the connectivity of various regions in the network is also different. Therefore, in order to parameterize the degree of reactivation of episodic association at a finer granularity, multiple-object tracking tasks with different difficulties are used to interfere with episodic memory [15]. In the case of different disturbances, the activation values of memory are also different. For example, in the case of think/no-think paradigm, the relationship between the differences in conditions and memory basically corresponds to the fact that there is no change in memory in the case of extremely low activation, while memory is weak in the case of moderate activation and enhanced in the case of high activation [16]. In the task with multiple-object tracking interference, subjects need to continuously track some moving target points during a period of time, while visualizing the scene associated with the words appearing in the center of the screen [17]. In this task, subjects need to be highly focused while tracking the targets; otherwise, the task will be difficult to complete successfully [15]. Studies have shown that such tasks related to visual working memory involve the parietal and frontal cortex. In addition, human cognitive resources are limited, and task performance is largely affected by the ability to selectively focus, memorize, and manipulate information according to task requirements [18]. The brain regions activated during this period overlapped with those of episodic memory to a certain extent, indicating that the activation of episodic memory and interference tasks would compete for visual resources. Therefore, studying this kind of episodic memory retrieval task that parameterizes the degree of memory activation can help to understand the conditions of episodic memory activation more comprehensively, and at the same time, from the perspective of the whole brain network, it helps to a broader understanding of the whole brain rather than focusing on the changes of the activation of certain regions; in this way, the coordination between network regions can be further considered from the specialization of regional functions.

In addition, word reading stimulates episodic memory retrieval in this task mode, the reading of English words will be affected by regions such as the temporal occipital and temporoparietal regions, and studies have shown that when reading English words, the brain activity and visual regions will have a strong coupling, English readers will have stronger activation of the subtemporal gyrus in tasks related to words retrieval [19]. Thus, the mentioned regions may have strong functional connectivity performance with the episodic memory circuit.

In order to explore the brain network model for the retrieval of disturbed episodic memory, a variety of methods were used in this study to try to construct a directed network in the task state, and the contribution of various regions involved in episodic memory as well as the broader coordination role of these regions was discussed from the perspective of network structure.

## 2. Materials and Methods

The fMRI data used in this study were obtained from the OpenfMRI database [17, 20]. The accession number of the data is ds002311, and the data are freely available at https://openfmri.org/data-set/ds002311/.

As shown in Figure 1, in this study, three methods of constructing brain function network using functional connectivity (FC) and effective connectivity (EC) were compared. FC matrices were calculated using Pearson correlation coefficient, and EC matrices were calculated using Granger causality analysis (GCA).

### 2.1. Participants

The original fMRI data set contains 23 right-handed T1 structural image data and four sets of functional image data [17]. The data of 8 of subjects was corrupted, so the data of the remaining 15 people were used. All were native English-speakers between 18 and 25 years of age with normal or corrected-to-normal vision and hearing.

### 2.2. Visual-Word Pairing Task Procedure

The whole experiment procedure is divided into six phases, and the fMRI data set contains the fMRI data from phase 3 to phase 6. This paper mainly studies phase 5.

Before phase 5 of the experiment, all the participants learned the 30 word-scene image pairs and performed a memory test to ensure that the participants remembered these pairs. At the same time, in order to control the situation of no visual association, before phase 5, each participant was shown 16 lure words without corresponding scene images. The participants were also required to be familiar with these lure words that appeared. These lure words will also appear in phase 5.

As shown in Figure 2, the subjects need to perform the targets tracking task for multiple times during phase 5, and try to reactivate the memory of word-scene image pairs in the procedure of targets tracking task interference. Before this, subjects had done similar targets tracking tasks many times to ensure that the subjects were familiar with the experimental procedure. In the target-tracking task, the subjects will see 10 random nonoverlapping points in the black background, among which the target points are red and the nontarget points are green (in the case of multitarget tracking, there are five target points, single target tracking with only one target point). There was a white fixation cross in the center of the screen. After a two-second exposure duration for subjects to memorize, all points were presented in green and began moving. Participants were asked to mentally track which points were originally the red target points for eighteen seconds. Meanwhile, the white central fixation cross was replaced by a word in white font with a small white dot in the center. If there was a scene image paired with the word (that is, the word was not a lure word), then the subject had to imagine the scene paired with the word in as much detail as possible. At the end of tracking, all points stop moving and one of the points turns white. The subjects need to select whether the white point is a target or a nontarget originally by pressing a button. After three seconds, participants were given feedback for one second indicating whether they were correct or incorrect. Finally, the participants completed two trails of an odd-even task: two numbers were displayed on the screen for 1.9 seconds, and participants need to press a button to determine whether the sum was odd or even. The text was presented in white, and when participants gave a correct response, the font was switched to green. When the response was incorrect, the font was switched to red. The interval between two odd-even tasks was 0.1 s, and after the two odd-even tasks, the screen was fixed for 4 seconds before the next multiple-object tracking task began. The total time of each trail of target tracking task was 32 seconds.

A total of 25 tasks were completed in a whole scan, among which there were 10 single-object tracking tasks of scene pairing words, 10 multiple-object tracking tasks of scene pairing words, and 5 multiple-object tracking tasks of lure words without pairing scene. The order of tasks was random. In phase 5, three fMRI scans were performed, with each subject performing a total of 75 tasks.

### 2.3. fMRI Data Acquisition

The MRI data were acquired by using a 3 Tesla whole-body Siemens Skyra MRI system. T1-weighted high-resolution MRI volumes were collected using a 3D MPRAGE pulse sequence optimized for gray-white matter segmentation, with slices collected in the AC-PC plane (176 sagittal slices; 1 mm thick; FOV = 256 mm; 256 × 256 matrix; TR = 2530 ms; TE = 3.37 ms; flip angle = 9°). The fMRI scans were collected using T2∗-weighted echo-planar image (EPI) acquisition (34 axial oblique slices; 3 mm thick; FOV = 192 mm; 64 × 64 matrix; TR = 2000 ms; TE = 33.0 ms; flip angle = 71°; 2 × IPAT acquisition).

### 2.4. Preprocessing of fMRI Data

Preprocessing of fMRI data was performed using the Statistical Parametric Mapping (SPM) Version 12 toolbox from Wellcome Trust Centre for Neuroimaging [21]. SPM provides a general method that can be adapted to most forms of experimental design and data analysis. It combines two mature theoretical frameworks (the general linear model and the theory of Gaussian fields) to provide a complete framework for the analysis of imaging data. This framework has conceptual and mathematical simplicity, and the generality of the framework provides for great latitude in experimental design and analysis. The preprocessing is divided into following steps. For each subject, the difference caused by different slice scanning time of each 3D image layer should be corrected at each time point, so that the whole brain image can be reconstructed accurately. In the process of slice timing, the middle layer of the 3D image is used as the reference layer. In the second step, we used the first scan in the time sequences as a reference image and aligned each image in the entire time sequences to the reference image, so as to correct the difference that the scanning images are not aligned due to the subject's head movement during the experiment. The functional image was spatially coregistered with the structural image and then used the EPI template to normalize the images and align the images to the Montreal Neurological Institute (MNI) Brain Template. In the original data, the voxel size is 3 × 3 × 3.9 mm, and the image dimension is 64 × 64 × 36, and the normalized image voxel size is 3 × 3 × 3 mm, and the image dimension is 61 × 73 × 61. Finally, a Gaussian kernel function of size 6 × 6 × 6 was used to smooth the image.

### 2.5. Functional Connectivity

Functional connectivity represents correlations between time sequences of different brain regions [22]. The correlation between two time sequences can be calculated by Pearson correlation coefficient:

(1) $$\begin{array}{c} \rho_{X,Y}=\frac{\text{Cov }\left(X,Y\right)}{\sigma_{X}\sigma_{Y}}=\frac{E\left(\left(X-\mu_{X}\right)\left(Y-\mu_{Y}\right)\right)}{\sigma_{X}\sigma_{Y}}, \end{array}$$

where *σ*_*X*_, *σ*_*Y*_ represent the standard deviation and Cov (*X*, *Y*) represents the covariance of the two time sequences. The range of *ρ*_*X*,*Y*_, the result of equation (1), is −1 ≤ *ρ*_*X*,*Y*_ ≤ 1. When 0 < *ρ*_*X*,*Y*_ ≤ 1, two time sequences show a positive correlation, and the greater the *ρ*_*X*,*Y*_ is, the stronger the positive correlation; when −1 ≤ *ρ*_*X*,*Y*_ < 0, two time sequences show a negative correlation, and the smaller the *ρ*_*X*,*Y*_ is, the stronger the negative correlation. *ρ*_*X*,*Y*_=0 represents that there is no correlation between two time sequences, that is, the two sequences are independent. This would reveal whether the two brain regions are functionally synergistic or antagonistic. In this study, the Brainnetome template [23] was used to divide the whole brain into 246 brain regions (excluding the cerebellum) according to anatomical structure. As shown in Figure 3, the time sequences of all voxels in each brain region were used to calculate the average time sequences, then we calculated the Pearson correlation coefficient of the average time sequences of each brain region in pairs. Thus, a 246 × 246 symmetric matrix was obtained, the value of each element in the matrix was the correlation of the brain region, and the rows and columns of the matrix corresponded to the number of brain regions. In order to obtain the FC matrix under three kinds of tasks, the average time sequences of each single task were extracted in this study. 25 tasks were performed on each scan, and 75 tasks were performed on three scans. However, the last task of each scan is incomplete, so these tasks were discarded, leaving 72 groups of average time sequences in total.

The FC matrix is a symmetric matrix calculated by the two time sequences, so the network structure represented by the matrix is undirected graph, so that there are some problems arise in the explanation of the network structure: when two time sequences *X* and *Y* show correlation, does *X* affect *Y*, or *Y* affects *X*, or does it affect each other, or are both *X* and *Y* affected by a third variable? Therefore, in order to eliminate these problems related to the direction of network, it is necessary to construct a model that considers causal influence, that is, effective connectivity.

### 2.6. Granger Causality Analysis

In 1969, Cliver Granger proposed the Granger causality analysis method [24]. It is defined as follows: for two stationary time series *X* and *Y*, if predicting the current value of *X* by the past value of *X* and *Y* is more accurate than predicting the current value of *X* by only using the past value of *X* itself, then *Y* is considered as the Granger cause of *X* [25]. This is implemented using a multivariate autoregressive (MVAR) model. In 1994, Friston applied GCA to neuroscience to obtain the EC between brain regions [26]. As a method of obtaining the EC matrix, GCA can build interaction mathematical models between different brain regions with statistically significant differences. The interaction between these brain regions can be used to infer the form of network connections. Consider the following autoregressive (AR) models:

(2) $$\begin{array}{c} X_{t}=\sum_{i=1}^{p}a_{1i}X_{t-i}+\varepsilon_{1t},\\ Y_{t}=\sum_{i=1}^{p}b_{1i}Y_{t-i}+\varepsilon_{2t}, \end{array}$$

where *a*_1*i*_ and *b*_1*i*_ are coefficients of the model, while *p* is the model order; that is, the current value is predicted using the previous 1 time point to the previous *p* time point. *ε*_1*t*_ and *ε*_2*t*_ are the residual errors, in the AR model of equation (2), *ε*_1*t*_ and *ε*_2*t*_ only depend on the past values of *X* and *Y*, and the accuracy of the model can be evaluated by the variance of the prediction error, namely, var(*ε*_*it*_), *i*=1,2.

Because *X* and *Y* may be affected by each other, *X* and *Y* are jointly considered to build a bivariate AR model:

(3) $$\begin{array}{c} X_{t}=\overset{p}{\underset{i=1}{\sum }}a_{2i}X_{t-i}+\overset{p}{\underset{i=1}{\sum }}c_{2i}Y_{t-i}+\varepsilon_{3t},\\ Y_{t}=\overset{p}{\underset{i=1}{\sum }}b_{2i}Y_{t-i}+\overset{p}{\underset{i=1}{\sum }}d_{2i}X_{t-i}+\varepsilon_{4t}. \end{array}$$

In the bivariate AR model, *ε*_3*t*_ and *ε*_4*t*_ are affected by both *X* and *Y*. For time series *X*, when the accuracy of the bivariate AR model is higher than that of the univariate AR model, that is, var(*ε*_3*t*_) < var(*ε*_1*t*_), then it can be said that *Y* causes *X*, and the causality measure is defined as

(4) $$\begin{array}{c} F_{Y⟶X}=\ln\left(\frac{\mathrm{var}\left(\varepsilon_{1t}\right)}{\mathrm{var}\left(\varepsilon_{3t}\right)}\right). \end{array}$$

When *F*_*Y*⟶*X*_ > 0, *Y* is the Granger cause of *X.* Similarly, the causal relationship from *X* to *Y* can also be obtained:

(5) $$\begin{array}{c} F_{X⟶Y}=\ln\left(\frac{\mathrm{var}\left(\varepsilon_{2t}\right)}{\mathrm{var}\left(\varepsilon_{4t}\right)}\right). \end{array}$$

As shown in Figure 4, using a method similar to the calculation of the FC matrix, the Granger causality matrix is calculated using the average time series of each brain area, that is, the EC matrix. The effect of causality is directed, *F*_*Y*⟶*X*_ and *F*_*X*⟶*Y*_ are not same, so unlike FC matrix, the EC matrix is not a symmetric matrix, and the network it represents is a directed graph. This would solve the FC influence direction problem mentioned in Section 2.5.

In this study, FC and EC were obtained by using time periods involving the reactivation of episodic memory, 0–18 seconds for each task. Because TR = 2 s, each time sequence only contains 9 time points, and the shorter length of time sequences also limits the choice of model order in GCA, so the first-order GCA model was used in this study.

### 2.7. Statistical Analysis

By analyzing the time sequence of each task, the FC matrix and the EC matrix were obtained. For the FC matrix, in order to be able to perform the group-level statistics, *Z*-score normalization should be performed for FC matrix of each task procedure to ensure that each sample has the same distribution. *Z*-score normalization is to find the difference between each variable and its mean divided by its standard deviation:

(6) $$\begin{array}{c} Z=\frac{X-\mu_{X}}{\sigma_{X}}. \end{array}$$

In this way, all the data are converted to the same distribution, with a mean of 0, and the standard deviation of 1. Then, the normalized FC matrices under the three task conditions can be averaged, respectively, to obtain the FC matrices in the three task states at the group level.

For the EC matrix, find the average EC matrix under the three task conditions. When the matrix element is greater than 0, there is causality between the two corresponding brain regions [25]. Therefore, using 0 as the threshold, connections with causality are selected and weighted directed network models under the three task conditions can be constructed, respectively. The weighted directed network is used to further construct the binary network when the word-scene image pairing memory is reactivated. In this process, the interference of the target tracking task added in the task design needs to be eliminated. In the multiple-object tracking task with pairing words, the episodic memory of the subjects was activated, as well as regions related to visual, motion, and target tracking tasks. Therefore, it was compared with the EC matrix of the multiple-object tracking task with lure words in this study. The EC matrices of these two task conditions were binarized. The elements of the EC matrix considered to have a causality are set to 1, and the elements that do not have a causality are set to 0. In this way, a binary network model in two task conditions was obtained. Keeping the connections that only appeared in the word-scene image pairing memory reactivation task but not in the lure word task, we can get the network related to episodic memory.

In addition, this study also used other methods to obtain binary EC matrices. The single-sample *t*-test was used for the results of GCA, and the connections with *p* < 0.05 were selected [27] to obtain the binary network of each sample. In order to obtain the binary network at the group level, the averages of connection numbers under the three task conditions were calculated for the binary network of each sample. The results are as follows: the average number of connections in the single-object tracking task with scene image pairing words is 5527 (standard deviation is 10.1669), the average number of connections in the multiple-object tracking task with scene image pairing words is 5469 (standard deviation is 10.3795), and the average number of connections in the multiple-object tracking task with lure words is 5408 (standard deviation is 6.0627). Add the binary matrices of the three task conditions respectively, and keep the connections that are shared by the most samples according to the average number of connections. For example, for a single-object tracking task with scene image pairing words, the top 5527 connections that are shared by the most samples are selected as the group-level result. For the other two task conditions, 5469 connections and 5408 connections are selected.

## 3. Results

Figure 5 shows the group-level FC under three task conditions. And Figure 6 shows the EC matrices under the three task conditions. Compared with FC, EC matrices in different conditions have more obvious differences, especially after binarization of the matrix. Therefore, the following discussion mainly focuses on the EC matrices.

In order to further analyze the differences between task states, the connections with causality are selected, the matrices are binarized, and the binary unweighted network is further analyzed. As shown in equations (4) and (5), if the *F* value of an element in an EC matrix is greater than zero, it means that the edge represented by this element has causal relationship. Therefore, with 0 as the threshold, the EC matrices under the three task conditions were binarized, and the binarized unweighted network represents a brain network model with causality. As shown in Figure 7, it is the EC matrices after binarization. There are certain differences in matrix elements under the three task conditions. It can be seen that compared with the single-object tracking task, a broader causal relationship appears in the multiple-object tracking task.

In order to control the influence of different task states on brain activity in the experiment, this study focuses on two multiple-object tracking tasks. These two task states have the same task requirements except for whether there is an episodic memory about word-scene pairs to reactivate. Although in the single-object tracking task, the simpler tracking task reduces interference and can stimulate the strongest reactivation under this condition, and it is difficult to compare with the lure word task as a control group due to too many different factors in the task. Although multiple-object tracking tasks cause weaker reactivation of episodic memory due to stronger interference, it is easier to control variables. Therefore, in this study, we subtracted the binary matrix of the multiple-object tracking task with pairing words and the binary matrix of the multiple-object tracking task with lure word. The different connections under the two task conditions were used to find out the differences in brain networks when episodic memory was activated or not, and the single-object tracking task that evoked the strongest episodic memory reactivation was used as a reference.

In this study, we also compared the binary EC matrices obtained by using the *t*-test to screen out elements with *p* < 0.05.  Figure 8 shows the connections shared by the most samples under the three task conditions, which are 5527, 5469, and 5408 connections, respectively. Since the EC network of a single sample after binarization has large differences between individuals, the number of shared connections is small (the connections with the highest share rate are only present in about 30% of the samples). This is difficult to be used as a basis for group-level analysis. Although there are some differences in the connections filtered according to the average number of connections, the reserved connections are too complicated, and the overall distribution still tends to be the same. It is difficult to determine whether these differences are decisive factors for different task states.

In summary, the most suitable method for analyzing the difference of network connection between the three states is to screen out the binarized EC matrices with *F* value greater than zero. In this study, BrainNet Viewer [28] was used to obtain the brain network.

Figures 9 and 10 show the episodic memory reactivation network obtained by using the pairing word task matrices to subtract the lure words task matrices. The complete connectivity matrix is uploaded to the supplementary material. It can be seen from the figure that the connections are mostly concentrated in the parietal lobe and the occipital lobe, and there is also a partial distribution in the prefrontal cortex. This is similar to the distribution of EC networks in single-object tracking. That means the brain networks obtained by subtraction are roughly similar to those when episodic memory activation is the strongest and with a small amount of interference.

The result indicates that the episodic memory brain networks obtained by this method are reliable. To further analyze the characteristics of the brain region connection, it is necessary to consider the direction of network edges. The brain network model obtained using this method is a directed unweighted graph, and as shown in Tables 1 and 2, the tables list all the indegrees and outdegrees of the brain gyri with causality.

Table 1 shows the indegrees of each gyrus in the binary network, that is, the number of connections with a certain gyrus as the end point. It can be seen from Table 1 that most of the edges end with medioventral occipital cortex and lateral occipital cortex, and there are also many edges with precuneus and fusiform as ends. Medioventral occipital cortex and lateral occipital cortex belong to the occipital cortex, which is closely related to vision [29]. In addition, studies have shown that the precuneus is involved in many advanced cognitive functions, including episodic memory [30, 31]. The fusiform is related to visual recognition functions such as semantic recognition and object recognition.

Table 2 shows the outdegrees of each gyri in the binary network, that is, the number of connections starting from a certain gyrus [32]. From Table 2, the starting points of most connections are concentrated on the superior parietal lobule, medioventral occipital cortex, and lateral occipital cortex. The superior parietal lobule is closely related to the occipital lobe, participating in attention and visual and spatial perception.

There are a total of 49 edges starting from the superior parietal lobule, of which 31 end in the medioventral occipital cortex and lateral occipital cortex, 7 end in the precuneus, and the rest are connected to the inferior temporal gyrus, thalamus, and parietal lobule. There are a total of 39 edges starting from the medioventral occipital cortex and lateral occipital cortex, of which 26 connect to the occipital lobe itself, and the rest connect to the regions such as the precuneus, fusiform, superior parietal lobule, and inferior temporal gyrus separately. The close synergy between the superior parietal lobule and the occipital lobe indicates that the reactivation of episodic memory produced by the superior parietal lobe can trigger the generation of visual imagination in the occipital lobe. The close connection between the temporal occipital, temporal parietal, and visual cortex plays an important role in the reading of English paired words [19, 33]. The connection of this part to the posterior parietal lobe indicates that the episodic memory is associated with the presence of the pairing word stimuli and activates the retrieval of the episodic memory.

## 4. Discussion

In this study, we compared and discussed various methods of constructing brain networks, and we constructed brain network models in word-visual association pairing tasks. The results showed that the posterior parietal cortex plays an important role in the episodic memory network. There is some debate about whether posterior parietal cortex is a memory region, but some studies have found that the region appears to be continuously involved in episodic memory retrieval [34]. From a dual-attention perspective, in the posterior parietal cortex, the superior parietal lobule and the intraparietal sulcus coordinate goal-oriented, “top-down” memory, while the inferior parietal lobule and the temporal parietal junction coordinate stimulus-oriented, “bottom-up” memory [32]. The posterior parietal cortex may be more closely associated with the representation of memory or as an input/output buffer for retrieval [35]. Studies have also shown that the parietal cortex is strongly activated in the encoding and retrieval of episodic memory [9], which is believed to be involved in the process of memory. In addition, there may be more detailed and diverse functional divisions in this part with low coupling, so there may be more facts to be explored in the functional study of this region [36, 37]. Consistent with most of the previous research results, the occipital lobe area as the visual center showed higher activity in tasks [29]. Many studies have mentioned that the precuneus, cingulate gyrus, orbitofrontal cortex, and prefrontal cortex play important roles in the circuit of episodic memory [31, 38]. In this study, the above regions show a high degree of causality, but the overall level of causality is inferior to that of the superior lobule and occipital lobe (medioventral occipital cortex and lateral occipital cortex). We speculate that the decrease in the overall activation level may be caused by the higher level of interference and the competition for resources between attention and situational recall, which is consistent with the presupposition in the multiple-object tracking experiment [39]. However, previous studies showed that some known memory regions in the medial temporal lobe, such as parahippocampal gyrus and hippocampus, are also involved in the process of episodic memory [40, 41]. These brain regions are also involved in the Papez circuit and default mode network, but these regions are not obviously involved in the network constructed in this study. There are only a few connections in the inferior temporal gyrus region. In general, the brain network model presented in this study is consistent with previous research results. Specifically, there are certain differences in the number and intensity of connections. This may be caused by different experimental designs and different interference intensities, which need to be further studied.

Studying brain networks related to episodic memory also has implications for disease diagnosis and pathology research. A study on PD has shown that the temporal lobe and parietal lobe of PD patients with mild cognitive impairment (PD-MCI) are atrophic, and the frontal cortex of patients is also thinner than the control group [42]. These regions have different levels of participation in the brain network constructed in this study. Episodic memory impairment is also common in the later stages of PD. A meta-analysis of 1,346 PD-MCIs from 8 different groups found that more than 50% of patients had memory impairment, while only 39% had executive dysfunction [43]. In addition, in the episodic memory task, the active regions of autistic patients and healthy individuals are similar, but the level of functional connection between the hippocampus and the frontal parietal region is weaker [5]. It can be seen from the above studies that some neurodegenerative diseases or other diseases such as autism may cause structural and functional changes in the episodic memory network and related brain regions.

From the results of this study, the network connectivity on the right hemisphere is denser than those on the left. Some previous studies have shown that in the encoding and retrieval process of episodic memory, many brain regions do not show obvious lateralization effect [34, 44, 45]. However, some studies have shown that in the retrieval of episodic memory, there are a wide range of brain regions showing left lateralization. From the perspective of microscopic neuron structure, there should be no significant differences between the left and right hemispheres of brain. However, when some disturbances occur during the memory encoding or retrieval process of the subjects, for example, different words or scenes presented in the memory process may cause certain emotions, which may cause the lateralization. This kind of result needs further analysis and discussion. Some data processing and statistical methods in the article also have room for further optimization. For example, since the EC matrix may be affected by some uncertainty or inaccuracy, there may be some noise that can interfere with the results. Some image processing-related methods may help to eliminate these inaccuracies, such as using some techniques based on fuzzy methods to process matrices [46, 47].

This study provides an idea of a method for constructing a task-based brain network model. From the brain network model, more complete information can be obtained than concentrated on a few brain regions, which is conducive to exploring the brain's changing pattern in the whole process. It helps to further understand the brain circuit related to episodic memory. At the same time, the study of brain network will help to further study about the disease from the perspective of whole brain function, including auxiliary diagnosis and targeted treatment measures.

Research on episodic memory helps humans to further understand the nature of the learning process. These studies have revealed different processes and different forms of memory production. Existing research can help people consider the complex interactions and wide-ranging effects of memory in a broader perspective in the future, help fundamentally determine the characteristics of human episodic memory, and interact with other advanced cognitive functions such as emotion, attention, and working memory. Because the task of the data set used is too complicated, the task focus may not be prominent, so only qualitative analysis is carried out in this study. In the future, we will consider the redesign of more focused experiments and conduct quantitative analysis, so as to further explore the clinical application of the study on episodic memory.

## Figures and Tables

**Figure 1:** Methods of constructing brain function network compared in this study. For FC, calculate and compare the group-level FC matrices under different task conditions, and try to construct a weighted undirected network; in order to further explore the direction of the network, use the GCA method to calculate the EC matrix, and build a network model based on the *F* value and *p* value, respectively.

**Figure 2:** The procedure of multiple-object tracking task.

**Figure 3:** The calculation of FC matrix. In this study, the whole brain was divided into 246 brain regions. Then, correlation coefficients were calculated in pairs. In this way, a 246 × 246 symmetric matrix was obtained. The matrix elements FC(*x*, *y*) and FC(*y*, *x*) represent the correlation coefficient between two brain regions of *x* and *y*. The paramaters *x* and *y* represent the indices of two brain regions in all 246.

**Figure 4:** The calculation of EC matrix. Similar to the calculation of the FC matrix, causality between brain regions was calculated in pairs and a 246 × 246 matrix was obtained. The matrix elements EC(*x*, *y*) represent the causal relationship from region *y* to region *x*. Also, the paramaters *x* and *y* represent the indices of two brain regions in all 246, as same as the indices in the FC matrix.

**Figure 5:** (a) FC matrix under single-object tracking task with pairing words; (b) FC matrix under multiple-object tracking task with pairing words; (c) FC matrix under multiple-object tracking task with lure words.

**Figure 6:** (a) EC matrix under single-object tracking task with pairing words; (b) EC matrix under multiple-object tracking task with pairing words; (c) EC matrix under multiple-object tracking task with lure words.

**Figure 7:** (a) Thresholded binary EC matrix under single-object tracking task with pairing words; (b) thresholded binary EC matrix under multiple-object tracking task with pairing words; (c) thresholded binary EC matrix under multiple-object tracking task with lure words.

**Figure 8:** (a) Binary EC matrix under single-object tracking task with pairing words, *p* < 0.05; (b) binary EC matrix under multiple-object tracking task with pairing words, *p* < 0.05; (c) binary EC matrix under multiple-object tracking task with lure words, *p* < 0.05.

**Figure 9:** The binary brain network model obtained by using GCA. The regions where the sum of the indegree and outdegree is greater than 3 are displayed. The size of nodes represents the number of degrees.

**Figure 10:** The connectivity matrix of the binary brain network obtained by using GCA.

**Table 1:** Indegrees of gyri.

Gyrus	Indegree of left or right hemisphere	Indegree of gyrus
Superior frontal gyrus	0 (L)	1
	1 (R)	

Middle frontal gyrus	0 (L)	2
	2 (R)	

Orbital gyrus	0 (L)	5
	5 (R)	

Paracentral lobule	1 (L)	1
	0 (R)	

Inferior temporal gyrus	2 (L)	7
	5 (R)	

Fusiform gyrus	7 (L)	10
	3 (R)	

Superior parietal lobule	0 (L)	4
	4 (R)	

Precuneus	10 (L)	15
	5 (R)	

Postcentral gyrus	3 (L)	4
	1 (R)	

Cingulate gyrus	2 (L)	2
	0 (R)	

Medioventral occipital cortex	14 (L)	36
	22 (R)	

Lateral occipital cortex	16 (L)	40
	18 (R)	

Thalamus	0 (L)	2
	2 (R)	

**Table 2:** Outdegrees of gyri.

Gyrus	Outdegree of left or right hemisphere	Outdegree of gyrus
Superior frontal gyrus	2 (L)	5
	3 (R)	

Middle frontal gyrus	1 (L)	4
	3 (R)	

Inferior frontal gyrus	0 (L)	1
	1 (R)	

Precentral gyrus	1 (L)	8
	7 (R)	

Fusiform gyrus	0 (L)	1
	1 (R)	

Superior parietal lobule	21 (L)	49
	28 (R)	

Inferior parietal lobule	0 (L)	7
	7 (R)	

Precuneus	3 (L)	7
	4 (R)	

Postcentral gyrus	0 (L)	1
	1 (R)	

Cingulate gyrus	1 (L)	1
	0 (R)	

Medioventral occipital cortex	7 (L)	15
	8 (R)	

Lateral occipital cortex	8 (L) 16 (R)	24

## Data Availability

The open dataset used in the article has been included and cited in the article.
